# Degradation of Toxic Dye Using Phytomediated Copper Nanoparticles and Its Free-Radical Scavenging Potential and Antimicrobial Activity against Environmental Pathogens

**DOI:** 10.1155/2021/1222908

**Published:** 2021-12-03

**Authors:** S. Rajeshkumar, M. Vanaja, Arunachalam Kalirajan

**Affiliations:** ^1^Nanobiomedicine Lab, Department of Pharmacology, Saveetha Dental College and Hospitals, Saveetha University, SIMATS, Chennai-600077, Tamil Nadu, India; ^2^SPKCES, Manonmaniam Sundaranar University, Alwarkurichi–627410, Tamil Nadu, India; ^3^Department of Science and Mathematics, School of Science, Engineering and Technology, Mulungushi University, Kabwe 80415, Zambia

## Abstract

The present investigation deals with the green synthesis of copper nanoparticles in an ecofriendly manner using leaf extract of *Andrographis paniculata*. Green-synthesized copper nanoparticles were studied for their antibacterial, antioxidant, and catalytic activity. The leaves were powdered and extracted with water and added to copper sulphate solution. The reduction of copper ions to nanoparticles was preliminarily identified by the color change of the reaction mixture. The synthesized nanoparticle was characterized by using a UV-Vis Spectrophotometer at a different wavelength with different time intervals. Functional groups available on the surface of the nanoparticle were identified by Fourier transform infrared spectroscopy (FTIR). Surface roughness was characterized by atomic force microscopy (AFM). X-ray diffraction (XRD) analysis showed six distinct intense peaks indicating the crystalline nature of synthesized copper nanoparticles (CuNPs). A scanning electron microscope (SEM) demonstrated polydispersed nanoparticles formed in the reaction process. The antibacterial activity of the nanoparticles was evaluated by an agar well diffusion assay against pathogenic bacteria. The antioxidant activity showed the excellent reduction of DPPH free radicals by nanoparticles. These results confirmed that copper nanoparticles serve as an alternative therapeutic agent over conventional drugs. Moreover, copper nanoparticles were also used to study the effect on the dye degradation process of methyl red and eosin dyes. Copper nanoparticles effectively remove the dyes with high efficiency up to 92% and 95% of methyl red and eosin dye, respectively.

## 1. Introduction

Nanotechnology creates nanomaterials with desired properties and small size falling into the nanometer scale [1]. The small-sized nanoparticles have a high surface area compared to bulk materials. Development of bioinspired nanoparticles is an immensely growing field in modern technology [2]. Various methods are available for fabrication of bioinspired nanoparticles such as physical, chemical, and biological methods. Moreover, the biological method includes using bacteria [3], fungi [4], virus and algae [5], and yeast and plants [6]. Microbe-mediated synthesis required frequent microbial cell culture maintenance and adequate handling experiences. But, among the methods, plant-derived nanoparticles are highly acceptable and preferable due to their environment friendliness, no usage of toxic chemicals, eliminating culture maintenance process, and no need of physical and chemical parameters [7]. Phytomediated synthesis of nanoparticles is based on the concept of phytoremediation of metals. Selection of plant for the nanoparticles synthesis is based on the heavy-metal resistance capability [8].

Among the noble metals, copper is abundantly available in the earth crust and exists in low stable metallic form. Copper is a crucial trace element in the biological system. Copper is extensively used because of high costs other noble metals compared to copper. Currently, copper nanoparticles have been attaining great attention due to their catalytic, optical, and electrical properties [9]. Therefore, copper is mostly preferred for the synthesis process because of low cost and high conductivity. Copper nanoparticles are widely used as antimicrobial, antioxidant, anticancer, anti-inflammatory, and antihepatotoxic agents. Currently, copper nanoparticles are used as an alternative feed additive in animal feed, especially poultry diet [10].

*Andrographis paniculata* (king of bitters) belongs to the family Acanthaceae, widely grown in Asian countries. In ancient medicinal system, this herb was used in therapeutic formulations to treat liver disorders. This plant has andrographolide, a bitter taste-giving major compound, and also has diterpene lactone [11] which is responsible for its pharmacological activities [12]. *A. paniculata* has various beneficial activities such as antioxidant [13], anticancer [14], hepatoprotective [15], antimicrobial [16], antidiabetic [17], antifertility [18], and antimalarial activity [19].

Methyl red is an azo dye with the molecular formula C_15_H_15_N_3_O_2_. Typically, methyl red dye is used in various industries such as textile, pharmaceutical, cosmetics, and tannery. The effluent releases from the industries are very toxic to the human beings.

The molecular formula of eosin is C_20_H_6_Br_4_Na_2_O_5_. Eosin is also commonly named as acid red 87, eosin yellowish, and so on. It is used for diverse purpose in the industries such as pharmaceutical, cosmetics, and textile. It is also used for tissue stain as well as counter stain. The existence of the hazardous dye in the terrestrial and aquatic environment leads to harmful health effects to the human beings such as cancer, tumor, and skin diseases.

In previous decades, physical and chemical methods were predominantly used for the degradation of dye. However, they have many draw backs. In order to avoid those issues, nowadays, biological methods are widely used for the degradation of hazardous dyes. Nowadays, nanoparticles are greatly receiving attention in degrading toxic dyes due to their large-surface-area properties [20]. In this study, copper nanoparticle was prepared by the simple green method and characterized. Synthesized nanoparticle was applied in various targeted applications such as antimicrobial, antioxidant, and catalytic activity.

## 2. Materials and Methods

### 2.1. Preparation of Plant Extract

The leaves of *A. paniculata* were collected from Vellore district. The freshly collected leaves were washed thoroughly with distilled water thrice and shade-dried for a few days at room temperature, and then, a fine powder was obtained using a blender. In this study, 5 g of plant powder was accurately weighed and added into a 250 mL conical flask containing 100 ml of double distilled water. The mixed suspension were boiled in a microwave oven for 5 minutes followed by double filtration accomplished with Whatman No.1 filter paper, and the consequent suspension was stored at 4°C for the further experiments.

### 2.2. Green Synthesis of Copper Nanoparticles

For the biosynthesis of CuNPs, 25 ml of aqueous leaf extract was assorted with 75 ml of distilled water containing 10 millimolar of copper sulphate. The prepared solutions were incubated in a shaker at room temperature for 24 h. After the incubation time, the change in the color of the solution owing to the formation of copper nanoparticles was observed by using a UV-Visible spectrophotometer.

### 2.3. Characterization of Green-Synthesized Copper Nanoparticles

Synthesis of copper nanoparticles was carried out by forming an SPR band measured in a double-beam UV-Vis Spectrophotometer. Crystalline structure and morphology of nanoparticles were observed by X-ray diffraction and scanning electron microscope analysis, respectively. The surface roughness and topography character were evaluated by atomic force microscopy analysis. Functional groups present on the surface of the nanoparticle were characterized by Fourier transform infrared spectroscopy.

### 2.4. Various Applications of Copper Nanoparticles

#### 2.4.1. Antibacterial Activity

Antibacterial activity of synthesized copper nanoparticles was determined by the agar well diffusion method. In this assay, about five microorganisms were used, *Bacillus* sp.*, E. coli, Klebsiella* sp.*, S. aureus*, and *Proteus* sp. Fresh overnight cultures of the abovementioned organisms were separately and evenly spread using a sterile cotton swab on a Muller Hinton Agar plate. About 6 mm diameter-sized four wells were made on the plate using gel puncture. Each well was filled with 50 *μ*L of leaf extract, 50 *μ*L (50 *μ*g/ml) of copper sulphate, 50 *μ*L (50 *μ*g) of copper nanoparticles, and 15 *μ*L (15 *μ*g) of standard (ampicillin). Plates were incubated at 28–30°C for 24 hours, and the zone formation around the well was measured.

#### 2.4.2. Antioxidant Activity (DPPH Scavenging Assay)

DPPH radical scavenging assay was performed using green-synthesized copper nanoparticles. DPPH solution was freshly prepared by mixing 0.004 g of DPPH in 95% methanol. 2.9 ml of DPPH solution was taken in four test tubes, and 0.1 ml of different concentrations (250–1000 *μ*g) of nanoparticles were added in each test tube. The reaction mixture was shaken vigorously and incubated for 30 min, and the resulting solution was measured at 517 nm in a UV-Vis spectrophotometer. Control was prepared containing the same concentration of standard ascorbic acid, and 95% methanol was used as blank. The scavenging property was calculated by using the following formula:

(1) $$\begin{array}{c} \%\text{inhibition}=\left[\frac{\left({\text{A}}_{\text{cont}}-{\text{A}}_{\text{test}}\right)}{{\text{A}}_{\text{cont}}}\right]\times 100, \end{array}$$

where A_cont_ is the absorbance of the control reaction and A_test_ is the absorbance in the presence of samples.

#### 2.4.3. Catalytic Reduction of Dyes

In this investigation, 10 mg of methyl red and eosin dye were prepared in 1 liter of double-distilled water in two conical flasks. From this stock solution, 100 mL of methyl red and eosin dye solutions were withdrawn and added into two conical flasks. 10 mg of green-synthesized copper nanoparticles was added into each conical flask, and control was maintained without addition of nanoparticles. The reaction solution was magnetically stirred and periodically measured by taking aliquots of 3 mL suspension and filtered. Filtered samples were monitored using a UV-Vis spectrophotometer at the wavelength from 300 nm to 800 nm.

## 3. Results and Discussion

### 3.1. Visual Observation and UV-Vis Spectroscopy Studies for Copper Nanoparticles

Preliminarily, synthesis of copper nanoparticles was observed by color change in the reaction mixture. Initially, the copper sulphate solution was in light blue color. Consequently, the color of the copper sulphate solution changes from light blue color to green on addition of leaf extract of *A. paniculata*, and eventually, dark greenish brown color was formed owing to the formation of CuNPs, as shown in Figure 1. The occurrence of the color changes in the aqueous solution is a result of the surface plasmon resonance phenomenon. The leaf extract of *A. paniculata* acts as a reducing agent as well as stabilizing agent, which reduced the copper sulphate into copper sulphide. The synthesis of copper nanoparticles was observed using UV-Vis spectra. The spectral readings for the concerned sample mixture were taken from 0 to 24 hours. Predominantly, the surface plasmon resonance of CuNPs exhibits the highest absorption peak at 530 nm, as displayed in Figure 2. Similarly, in previous studies, it has been reported that the surface resonance plasmon of CuNPs is in the range of 500–600 nm. On the other hand, it has been revealed in the range of 550–650 nm [21, 22].

### 3.2. FTIR Studies of Nanoparticles

The FTIR spectral study was carried out for the green-synthesized copper nanoparticles. The analysis was accomplished to find out the phytochemical constituents present in the crude extract of *A. paniculata*. These biomolecules act as a stabilizing and capping agent to bind with the metals. The peaks obtained in the copper nanoparticles are shown in Figure 3. The broad band at 3250.05 cm^−1^ ascribed to C-H stretching vibrations of alkynes, hydrogen-bonded O-H stretch of phenol, and alcohols. Furthermore, it also indicates the existence of N-H stretching vibration of secondary amine and the presence of N-H stretch of amide which is similar to the amine group. The IR band at 1730.15 cm^−1^ is attributed to the presence of organic compounds such as C = O stretch of ketones, C = O stretch of aldehydes, and C = O stretch of esters. The band examined at 1595.13 cm ^−1^ illustrates the corresponding aromatic compounds such as symmetrical C-C = C stretching vibration of aromatic rings, N-H bend of primary amines and amides, and the stretching vibrations N = O of nitro groups. The occurrence of band from 601.79–455.20 cm^−1^ exhibits the formation of copper nanoparticles [23]. The previous study also confirmed that the existence of band near 400–600 cm^−1^ indicates the formation of CuO [24]. The existence of phytochemicals in the crude extract of *A. paniculata* acts as a reducing and capping agent which has an ability to reduce the Cu2+ ion to copper nanoparticles.

### 3.3. AFM Studies of Nanoparticles

Atomic force microscopy was carried out to investigate about shape and features of the nanoparticles. The topography of the CuNPs was examined in the range of 2 *μ*m and 800 nm, as shown in Figure 4. The images show the spherical shape with doping of biomolecules on the surface of the synthesized copper nanoparticles.

### 3.4. XRD Studies of Nanoparticles

The X-ray diffractometer analysis was investigated to identify the crystalline nature of the synthesized copper nanoparticles (Figure 5). The diffraction peak of CuNPs exhibited at 2*θ* was found to be in the range of 20–40° which corresponds to the planes of (100), (002), (102), (103), (006), and (103). These planes indicate the crystalline formation of zinc sulphide nanoparticles. The average particle size of CuNPs was identified using the formula of Deybe–Scherrer. For CuNPs, the average size was 68 nm. As per the previous studies, it has been reported that the size of the copper nanoparticles ranges from 42–90 nm [9].

### 3.5. SEM Images of Nanoparticles

The SEM analysis was carried out for the green-synthesized nanoparticles and to identify the morphology structure of the particles.  Figure 6 shows the needle shape morphology to the nanoparticles. SEM image described polydispersed nanoparticles, particularly rod, spherical, and cube shape of nanoparticles with agglomeration.

### 3.6. Applications of Copper Nanoparticles

#### 3.6.1. Antibacterial Activity of Nanoparticles

In the present study, green-synthesized copper nanoparticles exhibited a predominant role against the pathogenic bacteria such as *S. aureus, Bacillus* sp.*, Proteus* sp.*, Klebsiella* sp.*, E. coli*, and *Pseudomonas* sp. by the well diffusion method. Four various control groups such as plant extract, precursor, and positive control (ampicillin) were used for the inhibition of pathogens, whereas the *A. paniculata*-mediated copper nanoparticles and precursor exhibit an excellent antibacterial activity against the test pathogens while compared to leaf extract and ampicillin, as depicted in Figures 7 and 8. This figure shows that *Pseudomonas* was inhibited by all the control groups. However, the CuNPs showed the maximum antibacterial activity against *Proteus* sp. followed by *Bacillus* sp.*, Klebsiella* sp., and *S. aureus*, and the minimum zone of inhibition was observed against *E. coli.* As per the previous study, it has been stated that the bactericidal property of copper nanoparticles is typically owing to the release of copper cations (Cu^+^ ions) and these copper cations are adhered to the cell wall of the bacteria owing to electrostatic attraction. Furthermore, the copper metal ions not only interact on the surface of a cell membrane but also perforate into the bacteria [21].

#### 3.6.2. Antioxidant Activity of Nanoparticles

The DPPH assay was performed to evaluate scavenging properties of the green-synthesized copper nanoparticles. The scavenging activities of CuNPs are identified owing to their ability of hydrogen donors. The result of various concentrations of CuNPs is shown in Figure 9. Ascorbic acid is used as a positive control. Results shows that both CuNPs and ascorbic acid exhibit the inhibition activity adjacent to the DPPH (1, 1-diphenyl-2-piciryl-hydrazyl) radicals. In the present study, the CuNPs exhibit the strongest inhibition of 53.04% at the concentration of 1000 *μ*g/ml. On the other hand, the positive control also shows the highest inhibition of 68.55% at the same concentration. Therefore, it implies that the scavenging activity of CuNPs increases while the concentration of the sample increases. The previous study also reported that the inhibitory activity increases when the concentration of the sample got increased. It also confirmed that the concerned sample exhibits higher antioxidant activity owing to the existence of phytoconstituents present in the crude extract [25].

#### 3.6.3. Catalytic Degradation of Methyl Red and Eosin Dye Using Nanoparticles

*(1) Mechanism of Catalytic Degradation*. As per the earlier studies, catalytic dye degradation was explained using the following mechanism. Catalytic reaction occurred on the surface of the metals present in the dye solution. Enhancing the surface area of the nanoparticles will also increase the efficiency of the catalyst used for the dye degradation. On the other hand, declining the size of the catalyst also enhances the catalytic reaction.

*(2) Catalytic Degradation of Methyl Red*. The catalytic activity of biosynthesized copper nanoparticles was determined by the reduction of methyl red dye at various intervals of time from 30 min–48 h. Initially, the reduction of dye concentration in a solution by using copper nanoparticles was observed by color change. The color of the dye solution changed from red to pale white indicates the degradation or removal of dye. The progress of the dye degradation was recorded using an Ultraviolet-Visible spectrophotometer in the range of 300–800 nm. In each interval, the maximum absorption peak was monitored at 415 nm for synthesized nanoparticles. Subsequently, the peak has been decreased gradually with the increase of time, which reveals the degradation of methyl red through the catalytic activity of the synthesized copper nanoparticles. The previous study also supported the result of the current study. However, in the former study, they used AgNPs as a photocatalyst for the degradation of methyl red dye [26].  Figure 10 shows that the peak at the time interval of 48 hrs was gradually declined when compared to the other time intervals. From this, it has been revealed that a green-synthesized copper nanoparticle has an ability to degrade the methyl red dye.

*(3) Catalytic Degradation of Eosin Dye*. The catalytic activity of the biosynthesized copper nanoparticles was investigated against the water containing eosin dye. The kinetic reaction was observed using the UV-Visible spectrophotometer technique in the wavelength of 300–800 nm.  Figure 11 shows that the maximum peak value was obtained in the range of 500–515 nm. As per the previous study, it also reported that the absorption spectrum of eosin was recorded at 517 nm [27]. Gradually, the peak disappears when the reaction time increases. Therefore, it indicates that eosin dye has been degraded in the existence of copper nanoparticles, as depicted in the figure.

## 4. Conclusions

Phytomediated synthesis of copper nanoparticles is a simple and ecofriendly method. In this study, plant leaf powder was used to prepare aqueous extract which was mixed with copper sulphate solution. The extract was reduced to copper sulphate and into copper nanoparticles. Synthesized copper nanoparticles were characterized by positioning of SPR band confirmed using UV-Vis Spectra. The crystalline structure and morphological characters were identified using XRD and SEM analysis. AFM image shows that topography characters of green-synthesized copper nanoparticles. The functional groups involved in the reduction of copper sulphate to copper nanoparticles were characterized by FTIR spectrum analysis. Hence, the synthesized nanoparticle was studied for medical applications such as antibacterial and antioxidant activity against pathogenic microorganisms and DPPH free radical. Other than that, the synthesized nanoparticle was utilized in environmental applications such as the toxic dye degradation process.

## Figures and Tables

**Figure 1:** Visual observation of synthesis of copper nanoparticles. (a) Leaf extract, (b) copper sulphate, and (c) final color of CuNPs was obtained after the synthesis process of completion.

**Figure 2:** UV-Visible spectra of copper nanoparticles measured at wavelength ranges from 300 nm to 800 nm.

**Figure 3:** FT-IR spectrum of green-synthesized copper nanoparticles.

**Figure 4:** Atomic force microscopy images of copper nanoparticles. (a) 2 *μ*m and (b) 800 nm.

**Figure 5:** X-ray diffraction spectrum of green-synthesized copper nanoparticles shows crystalline structure.

**Figure 6:** Scanning electron microscopic images of copper nanoparticles synthesized using *A. paniculata*.

**Figure 7:** Antibacterial activity of copper nanoparticles. (a) *Proteus*, (b) *S. aureus*, (c) *Klebsiella*, (d) *Pseudomonas*, (e) *E. coli*, and (f) *Bacillus* sp.

**Figure 8:** Graphical representation of the antibacterial activity of copper nanoparticles. *Y*-axis: zone of inhibition in mm, and *X*-axis: bacterial pathogens.

**Figure 9:** Antioxidant activity of copper nanoparticles against DPPH free radical. *Y*-axis: percentage of inhibition in mm, and *X*-axis: concentration of nanoparticles.

**Figure 10:** Catalytic degradation of methyl red using copper nanoparticles. *Y*-axis: absorbance, and *X*-axis: wavelength in nm.

**Figure 11:** Catalytic degradation of eosin using copper nanoparticles. *Y*-axis: absorbance, and *X*-axis: wavelength in nm.

## Data Availability

The data used to support the findings of this study are included within the article.
